The article "Al2O3/ZrO2 dual-dielectric Gr/CNT nanoribbon vertical tunnel FET based biosensor for genomic classification and S-protein detection in SARS-CoV-2" was retracted in 2025. Reasons: unreliable results or conclusions; concerns about the citations.

# Al_2_O_3_/ZrO_2_ dual-dielectric Gr/CNT nanoribbon vertical tunnel FET based biosensor for genomic classification and S-protein detection in SARS-CoV-2

**DOI:** 10.1016/j.heliyon.2024.e30077

**Published:** 2024-04-24

**Authors:** M. Venkatesh, P. Parthasarathy

**Affiliations:** Department of Electronics and Communication Engineering, CMR Institute of Technology, Bengaluru, Karnataka, India, 560037

**Keywords:** SARS-CoV-2, Biosensor, Charge density, Genomic behaviour, Mutation, Dielectric behaviour

## Abstract

The ongoing genetic mutation of severe acute respiratory syndrome coronavirus 2 (SARS-CoV-2) possesses the capacity to inadvertently lead to an increase in both the rates of transmission and mortality. In this study, we showcase the use of an Al2O3/ZrO2 Dual-Dielectric Gr/CNT Nanoribbon vertical tunnel field-effect transistor biosensor for the purpose of detecting spike proteins of SARS-CoV-2 in clinical samples. The proteins mentioned above are situated within the protein capsids of the virus. The effectiveness of the suggested detector has been assessed through measurements of the alteration in current drain. The present study utilizes the dielectric coefficient analogue of viral proteins as a substitute for biomolecules that exhibit internal hybridization nanogaps. The high sensitivity of the suggested detector, as evaluated on a scale ranging from 0 to 115, suggests its potential as a high-quality sensing instrument. The purpose of this study is to examine the sensitivity of DNA charge density with the aim of identifying any alterations in the virus that may impact its ability to spread and infect humans. The chromosomal composition of SARS-CoV-2 has been determined. The CMC Research Centre, situated in Vellore, Tamil Nadu, India, conducted an examination of SARS-CoV-2 samples. The scientists possess the capability to do genome sequencing on these specimens, so facilitating the examination of mutation patterns and the dispersion of different clades. A total of 250 different mutations were found out of the 600 sequences that were evaluated. The sequencing data consists of a complete collection of 250 distinct variants, including 150 missense mutations, 80 synonymous mutations, 15 mutations in noncoding regions, and 5 deletions. The comprehension of genetic variety is significantly dependent on these mutations. The proposed detector is connected to a variety of previously documented biosensors based on field-effect transistors (FETs), which are employed for the examination of genetic modifications.

## 1 Introduction

The family of coronaviruses is responsible for a wide range of respiratory illnesses in humans. The initial identification of human cases of SARS-CoV-2 (severe acute respiratory syndrome coronavirus 2) occurred in Wuhan City, China, around the mid-2019 period. The respiratory coronavirus that developed in 2019 was designated with the name "COVID-19." The World Health Organisation classified it as a pandemic on March 11, 2020 [1,2]. The first instance of SARS-CoV2 was identified in a Turkish individual who had recently returned from Europe on March 11, 2020. The first recorded death occurred on March 17. Following the initial diagnosis, the pandemic has rapidly spread worldwide, even within the borders of Turkey. The Indian Ministry of Health recorded around 400,000 deaths and one million instances of illness as of June 2021. Various initiatives have been implemented globally to address the rising prevalence of public health concerns [3]. The COVID-19 pandemic necessitated a reorganization of virology laboratories in order to enhance the efficiency of viral detection. Several laboratory diagnostic approaches, including real-time polymerase chain reaction (PCR), quick antibody, and Immunosorbent Assay Enzyme-Linked, have facilitated the prompt and precise diagnosis of COVID-19. The RNA virus of SARS-associated coronavirus 2 (CoV2) is undergoing continuous evolutionary changes. According to reports, there have been mutations in the genome of the virus, potentially leading to an increase in both the transmission rate of the sickness and the number of fatalities it causes. To comprehend the origins, methods of transmission, and mutations that affect the pathogenicity of SARS-CoV2, it is essential to classify the full-length SARS-CoV2 sequences at the molecular level. The research of genetic sequence data also holds substantial potential for the advancement of novel medications and vaccines [[4], [5], [6]]. The emergence and rapid dissemination of novel SARSCoV2 subtypes were observed during the COVID-19 epidemic. Fig. 1 illustrates the whole configuration of Covid-2, which consists of two proteins: spike and Nucleocapsid. Scholars have conducted investigations into the proliferation of viruses by the analysis of their genetic variants, enabling the identification of novel strains and their interconnections. The molecular epidemiology of SARS-CoV2 has been monitored through the utilization of internet sequence-sharing technologies and the accessibility of freely available virus genome sequences.

**Fig. 1:** General schematic of Covid-2 with spike protein and Nucleocapsid protein [6].

Multiple research efforts conducted during the epidemic examined the genomic characteristics and phylogenetic connections of SARSCoV2 genomes that were circulating worldwide. On March 25, 2020, Turkey submitted the initial genome sequence of SARSCoV2 to the Global Initiative on Sharing All Influenza Data (GISAID). Subsequently, by May 31, 2021, Turkey had contributed over 4000 sequences to the initiative. The molecular characterisation and phylogenetic analysis techniques were employed to trace the origin of the initial comprehensive SARS-CoV2 genomes to Europe. The genomes of SARS-CoV-2 were isolated and sequenced in Turkey, indicating that the country was the first to be infected with the virus. The genomes of SARS-CoV-2 in Turkey have been the subject of studies [7,8], which have revealed the virus's capacity to undergo various nucleotide modifications, including both silent and missense mutations, since the onset of the pandemic. The presence of SARSCoV2 genomes in Turkey is observed across many lineages, as delineated by naming systems. The virus diversity data of the country indicate the origins from which the virus has disseminated to multiple sources and subsequently undergone adaptation to its novel environment. The ELISA test is not intended for viral identification, but rather for the detection of particular antibodies present in the blood serum of the patient. The current gold standard for diagnosis is real-time RT-PCR, which detects the E-protein RNA (N-Protein), open frame reading b1 (OFRb1), and OFRb2 genes from a nasal swab. The process of virus identification commences by inserting a single sample of viral RNA into a designated testing kit. Following this, a primer is introduced to the viral RNA in order to enhance the process of replication. The protein Spike on SARS-CoV and SARS-CoV-2, as well as the host cell, is depicted in Fig. 2. The activities of the protein are described in the sources [9,10], illustrating the S1-ECD domain protein Spike in Fig. 3 and the S2-ECD region in Fig. 4. Furthermore, the RNA of the virus undergoes synthesis to form complementary DNA (cDNA), which is then duplicated through the process of DNA polymerization. Complementary DNA (CDNA) is a term used to describe synthetic DNA that possesses a base sequence that is complementary to a pre-existing DNA sequence. CDNA synthesis necessitates the utilization of RNA as a template. Upon reaching a specific temperature, the DNA undergoes denaturation, resulting in the separation of the two strands. Following the denaturation of the DNA helix, the primer, fluorescent reporter molecules, and quencher are subsequently annealed and included as a component of the probe. SARS-CoV2 RNA virus exhibits frequent variation. The accumulation of new mutations in the genome of SARS-CoV2 will lead to an increase in transmission and fatality rates, as supported by arguments [11,12].

**Fig. 2:** SARS-CoV & SARS-CoV-2 with Anheftungsprotein Spike and host cell [13].

**Fig. 3:** SARS CoV-2 Spike Protein Schematic with a wide range of high-affinity Spike/ECD rabbit mAbs span the S1-ECD and the S2-ECD region of the Spike protein [14].

**Fig. 4:** Schematic overview of the SARS-CoV-2 Spike (S) protein and its functional domains [15].

This study investigates the electrical conductivity of the S-protein of SARS-CoV-2 in order to enhance the development of a TFET-based biosensor for the diagnosis of SARS-CoV-2 and the schematic overview of the SARS-CoV-2 Spike (S) protein and its functional domain is depicted in the above Fig. 4. The glycoprotein S-protein of COVID-19 has a dielectric constant ranging from around 1 to 4, similar to that of biotin-streptavidin. The electrical conductivity of DNA, as documented in scientific literature, ranges from 1 to 64. A unique approach to virus detection involves the utilization of S-protein, which converts viral RNA into C-DNA. This study aims to analyze and contrast the sensitivities of several TFET-based biosensors that have been reported in the literature for the detection of SARS-CoV-2 [14,15]. We suggest utilizing the vertical Tunnel FET as the foundation for a biosensor due to its distinctive steeper subthreshold swing characteristics, faster switching, and quantum mechanical tunnelling-based operation. The unique characteristic of VTFETs is responsible for their extraordinary sensitivity in sensing applications. The process of sensing occurs within nanogaps that are formed with the removal of a portion of the oxide layer, resulting in the immobilization of the target molecules. The building of the gate incorporates both iron and steel materials. This minimizes the likelihood of the target molecules undergoing chemically significant alterations due to their reactivity with the ionic liquid gate solution. Furthermore, this study examines the mutation profile by sequencing the complete genome of SARS-CoV2 positive samples that were evaluated in our laboratory. The subsequent section provides a concise summary of the phylogenetic analysis and mutation pattern observed inside the genome. In order to gain a deeper understanding of the phylogenetic context and genomic diversity of the isolates from a global perspective [[16], [17], [18]], we calculate the distribution of clades using three naming systems: Pango lineage, Nextstrain, and GISAID.

## 2 Severe acute respiratory syndrome coronavirus 2 biosensors

The late 2019 coronavirus containment blamed for severe acute respiratory syndrome (SARS-CoV-2) occurred in Hubei Province, China. The COVID-19 outbreak, which was officially proclaimed by the World Health Organisation (WHO) in 2020, has resulted in the infection of more than 20 million individuals and the unfortunate loss of over 800,000 lives. The repercussions of this phenomenon have permeated across the economy, eliciting concerns among certain individuals on the potential occurrence of a financial collapse and following economic downturn. An infectious viral outbreak poses a significant threat to both public health and the global economy. The 2009–2010 Influenza (H1N1) epidemic, the ongoing global HIV epidemic, the Ebola outbreak and epidemic (expected to persist until 2020), the Zika epidemic (occurring in 2015–2016), and the current COVID-19 outbreak are among the notable instances of recent global health emergencies. Treatment or immunization for outbreak-causing viruses is seldom [[19], [20], [21], [22]]. Mass testing is conducted to identify epidemics in order to locate contacts and prevent the propagation of the disease. Consequently, the reduction of infection rates and cessation of virus transmission can be achieved by the utilization of a prompt, precise, and reliable diagnostic process. Common diagnostic procedures include polymerase chain reaction, enzyme-linked immunosorbent tests, and Western blotting for viral cultivation-based diagnostics. Nevertheless, due to the exorbitant expenses and intricate nature of the requisite research laboratory apparatus and personnel, these approaches are suboptimal for expeditious on-site assessment. Prompt identification is not always feasible, and the protocols can be protracted. Consequently, the implementation of mass testing, which is crucial during pandemics when time is of the essence, becomes more challenging. Therefore, there is a need for a prompt, highly responsive, and precise point-of-care (POC) device that can be utilized in clinical environments or at home [23].

Given the potential advantages offered by biosensors, it is crucial to undertake additional research and development in this field. A biosensor refers to a form of analytical apparatus that ascertains the concentration of an analyte by utilizing the signal generated by a biological process. The individual components of a bioreceptor include a transducer and a reading device. Bioreceptors have been developed in order to identify and respond to a particular target analyte [23]. The utilization of biosensors may encounter logistical limitations due to factors such as storage duration (shelf life), operational time, or longevity. The longevity of a biosensor can vary from a few days to a few weeks, contingent upon elements such as the receptor's stability and the conditions of storage and operation. Nevertheless, it is anticipated that commercial biosensors would possess a storage duration ranging from six months to one year [23]. Enzymes and their substrates, antibodies and their targets, or complementary nucleic acid systems can carry out bio-affinity and biocatalytic tasks, depending on the analyte and the bioreceptor. Various types of transducers, including as electrochemical, optical, thermal, and piezoelectric transducers, can be employed to convert the interaction between a bioreceptor and an analyte into a readily detectable signal. The observed phenomenon can be construed as an identifiable electrical signal within the context of electrochemical biosensors. Over the past decade, a significant proliferation of electrochemical biosensors capable of detecting proteins, cancer biomarkers, viruses, and bacteria has been observed. The utilization of immobilized forms of antibodies, antigens, or nucleic acids was observed in the majority of virus detection receptors [23]. In 1962, Clark and Lyons successfully developed the inaugural electrochemical biosensor by employing the enzyme glucose oxidase. The oxygen electrode was coated with glucose oxidase and placed behind a selectively permeable membrane, facilitating the passage of glucose. The magnitude of the signal exhibited a clear correlation with the rate of oxygen consumption. Following this specific time frame, Adam Heller improved the detection of glucose and obtained patents for multiple concepts related to electrochemical biosensors in order to safeguard his advancements. The gold standard consists of affordable biosensors that exhibit exceptional sensitivity and specificity. Electrochemical biosensors are advantageous due to several reasons: (i) the cost-effectiveness of microelectronic circuits and their seamless integration with standard electronic readouts, (ii) the reliability and user-friendly nature of electrochemical biosensors, (iii) their compact size and compatibility with microfluidic devices, and (iv) the superior accuracy of electrochemical biosensing compared to alternative biosensor design methods like optical, piezoelectric, and microbalance.

However, the production of electrochemical biosensors necessitates meticulous deliberation of many components, akin to the advancement of any other type of biosensor. The operational efficacy and durability of biosensors are contingent upon the biocompatibility of the materials employed in their fabrication. For the bioreceptor to effectively bind to the analyte, it is imperative that the immobilization matrix concurrently provides protection to the bioreceptor against potentially detrimental environmental factors, including alterations in pH, ionic strength, and temperature. Table 1 provides the same with Synopsis of SARS-CoV-2, Zika, HIV, Influenza and Ebola Biosensor Performance Characteristics. The enhanced sensitivity and improved detection capabilities of biosensors can be attributed to advancements in immobilization techniques and the utilization of materials such as conducting polymers and nanoparticles. Nanotechnology has greatly advanced electrochemical biosensing in recent decades, offering a convenient and effective method for monitoring analyte concentrations and diagnosing diseases [24].

**Table 1:** Synopsis of SARS-CoV-2, Zika, HIV, influenza and ebola biosensor performance characteristics.

Virus	Element - Target	Element - Recognition	Method of Detection	Detection Limit	Working Range	Ref
Influenza - the flu	Antibody/RGO/Cystamine	Modified GCE	CA & CV	0.7 PFU/mL	2.0–105 PFU/mL	3–4
H9N_2_ - Influenza	NA	Hybrid Nanocomposite with GR/CNT	EIS - SPE	10.0−8.0 U/mL	11.0−9.0 to 11.0−2.0 U/mL	5
H9N_2_ - Influenza	Protein Fetuin-matrix	AuNPs with matrix-based composite	CV & CVP	20 HAU	9.0–127.0 HAU	6–7
H1N1/H1N5 HA - Influenza	GO/Methylene Blue/Chitosan-protein A/Antibody	Screen Printed Electrode	DPV	8.5 pM	26.0−600.0 pM	8
Influenza	Anti-H5 HA - Antibodies	His6 -H5 HA/DPM-Cu (II)	SWV	2.5 pg/mL	5.5–106.0 pg/mL	9
HIV	Anti-HIV p24 - Antibody-based	SPE with Single walled CNT	DPV	2 pM	11 pM to 2 nM	10
HIV	Antibody-based on Anti-HIV p17	LBL to immobilize Lignin	EIS	–	1.5 nM–106 nM	11
HIV	Liquid ion gate-FET	Viral DNA	FET	0.5 aM	11.0−19.0 to 11.0−9.0 M	12
HIV	Viral Genome	rGO/CNT	Electron Impedance Spectroscopy	0.3 pM	16−19 to 17−20 M	13
HIV	DNA - Viral	DNA Probes with Nanocluster/GCE	Differential Pulse Voltammetry	3 × 10−17 M	11−17 to 11−12 M	14
Ebola	Viral Glycoprotein	Antibody/rGO-FET	Field Effect Transistor	2.5 pM	3.5 pM to 25 μM	15
Ebola	Viral cDNA	cDNA probe/Au-SPE	Differential Pulse Voltammetry and Electron Impedance Spectroscopy	5.0 nM	11.0–90.0 nM	16
Zika CV	NS1	Antibody/Cystamine/GAZnO nanostructure-print circuit board	Cyclic Voltammetry	Less than 3.0 pM	–	17
SARS-CoV-	Spike Protein	SpAb/AuNPs/FDTO	Differential Pulse Voltammetry	–	–	18
SARS-CoV-2	Spike Protein	SpAb-PBASE/Graphene-FET	Field Effect Transistor	17 pfu/mL	–	19–20

Due to its advancements, electrochemical biosensors are widely used in point-of-care diagnostic equipment. This project aims to construct biosensors using layered dielectric TFETs for sensitive SARS-CoV-2 antigen detection. An outbreak has broken out due to this virus. Protein identification and genome sequencing and characterization were the main goals of this project.

## 3 Methodology

### 3.1 Simulation strategy and device structure

The SARS-CoV-2 biosensor depicted in Fig. 5 is constructed using an Al2O_3_/ZrO_2_ Dual-Dielectric Gr/CNT Nanoribbon Vertical Tunnel FET. This 2D structure has been specifically designed to enhance the detection capabilities of SARS-CoV-2. The device exhibits both horizontal and vertical tunnelling capabilities due to the presence of a 20 % doped pocket in SiGe. The N pocket consistently exhibits a doping concentration of $1.3\times 10^{18\;}{cm}^{-3}$ in many studies. Fig. 5 displays the measurements for the gadget. This sensor design utilizes two metal gates with energies of $\varphi_{M1}=4.4\;ev$ (Source side) and $\varphi_{M2}=4.5\;ev$ (drain side) to optimize the I_ON_/IO_FF_ ratio. The doping concentrations exhibit a range of $1.1\times 10^{20\;}{cm}^{-3}$ in the source region to $5.1\times 10^{18\;}{cm}^{-3}$ in the channel region to $2\times 10^{18\;}{cm}^{-3}$ in the drain region. The fixed dual dielectric material Al2O_3_/ZrO_2_ possesses a length of 15 nm. The architecture incorporates a 2 nm thick Al_2_O_3_ layer to immobilize receptor molecules and reduce leakage current. Sensing takes place in an entirely arid environment under this situation. In Silvaco Atlas, each simulation is executed.

**Fig. 5:** 2D schematic of a Graphene channel Ge-source dual dielectric Vertical TFET (VTFET)-based bio-sensor.

The device-level BTBT mechanism uses non-local BTBT. According to the bandgap narrowing theory, the simulation reduces the forbidden energy bandgap. This narrowing is caused by increased doping in the drain and source areas of the device. The SRH hypothesis is employed to elucidate the mechanism by which indirect bandgap materials induce recombination. The key mechanism behind the operation of this type of biosensor is the coupling between the gate and the channel. The incubation of biomolecules within cavities leads to an elevation in the effective gate capacitance, hence causing an augmentation in the coupling between the cavities in comparison to an empty state. This phenomenon results in an increased drain current due to the concentration of a larger quantity of electrons within the channel, surpassing the typical scenario. During the simulation process, an insulator with an identical dielectric constant to the biomolecule of interest is employed as a substitute. This facilitates the attainment of the intended outcome [24]. This insulator completely occupies all of the vacant areas. With 1k, voids insulate like air. VFET-based dual dielectric modulated graphene channel Ge source biosensors have been shown to be feasible in various investigations. The vertical TFET-based COVID-19 sensor's suggested detection mechanism is shown in Fig. 6.

**Fig. 6:** Detection Process of the proposed vertical TFET biosensor.

### 3.2 Device fabrication & characterization

The vertical TFET structure was produced using a top-down technique, which involved epitaxial growth of an n-type doped layer on a (100) n-type bulk Si substrate with 1 × 10^19^ arsenic atoms. The differentiation between functional and non-functional regions is achieved through a local oxidation process (LOCOS). In areas characterized by active growth, the Si layer is utilized to cultivate a vertical structure. Subsequently, a conformal layer consisting of 1 nm Al_2_O_3_ and 1 nm ZrO_2_ is applied onto the Si substrate, resulting in the formation of a double gate stack that encircles the edges of the device, specifically the oxide layer situated between the stack and the substrate. Subsequently, chemical mechanical polishing (CMP) is employed to enhance the surface quality following the application of an oxide coating. When the oxide and gate stack are etched away, the upper section becomes exposed, leading to a gate length of around 70 nm. The process of ion implantation results in the formation of a top junction that exhibits inherent alignment with the gate, while the dual gate layer extends by a further 80 nm beyond the threshold and the same has been depicted in Fig. 7a.

**Fig. 7:** a Device fabrication process: An Overview, b displays a high-resolution scanning TEM (STEM) image of the vertical TFET, demonstrating the dry transfer process's clean interface.

## 4 Results and discussion

### 4.1 Charge sensitivity analysis for neutral state

Fig. 7b displays a high-resolution scanning TEM (STEM) image of the vertical TFET, demonstrating the dry transfer process's clean interface and Fig. 8 shows VTFET-based sensor ID-VGS characteristics for different dielectric constants (k). This investigation assumes that viral protein and C-DNA are neutral. The drain current exhibits a decrease in the absence of biomolecules, while it demonstrates an increase in the presence of biomolecules and the filling of nanogaps (k = 1.2, 2.84, 6.33, 8.46). Once the nanogaps have been filled by biomolecules, the drain current will increase. The significant change in channel conductivity occurs as the effective gate capacitance increases, leading to the hybridization of biomolecules produced by the immobilized receptors enclosed within the nanogaps [25,26]. Effective gate capacitance quantifies the extent to which a gate is actively conducting.

(1) $$C_{eff}=\frac{E_{Bio}E_{{ZrO}_{2}}}{E_{Bio}T_{{ZrO}_{2}}+E_{{ZrO}_{2}}T_{Bio}}$$

**Fig. 8:** Transfer properties of a label-free vertical TFET biosensor for SARS-CoV-2 detection.

Assuming complete filling of all nanogaps, the symbol C_eff_ can be employed to determine the effective capacitance per unit area. Based on Equation (1), it may be inferred that the value of C_eff_ increases proportionally with the increase in e_bio_ (the number of k).

The increasing number of electric field lines will cause charges to accumulate in the channel region. Thus, drain current increases significantly. Fig. 9a and b shows biomolecules' horizontal and vertical energy band diagrams for different k values. Band bending is stronger at k = 8.46, which makes drain current vary more than at other k values [26]. The SARS-CoV-2 sensor's drain current sensitivity is tested in the state k = 1 (air), which reflects the nanogaps' absence of substances.

**Fig. 9:** a& 9b. Energy distribution in the conduction and valence bands along horizontal and vertical axes for various k values and orientations.

The sensitivity is measured using Equation (2),

(2) $$S_{N}=\frac{I_{K,Dr}}{I_{Air\;\left(K=1\right),Dr}}\left(\text{At}\;\text{fixed}\;\text{gate}\;\text{voltage}\;\text{and}\;\text{drain}\;\text{voltage}\right)$$

$I_{K,Dr}$ and ${\;I}_{Air\;\left(K=1\right),Dr}$ represent the drain current at a fixed gate (V_GS_) and drain voltage (V_DS_) for filled (S-proteins or C-DNA) and empty nanogaps.

Fig. 10a illustrates the drain current sensitivity map for the three proteins with neutral charges that were considered. Due to the inclusion of the Ge Source at the junction between the source and channel, this specific device exhibits a sensitivity of approximately 110 at k = 8.46, surpassing the sensitivity of previous devices. This illustrates that in comparison to other biosensor types, this particular one exhibits a greater degree of feasibility. The reaction time for the proposed biosensor is defined as the duration required for the measured value to exhibit a 90 % rise from the initial point of input change in the variable. The duration is ascertained by commencing from the moment when the alteration in the variable's step input commenced. Fig. 10b clearly demonstrates that the response time is a mere 10 ps, positioning it as one of the most rapid in the business. The vertical TFET exhibits a more pronounced sub-threshold swing compared to the horizontal TFET. The rationale behind this is that vertical TFETs are positioned in a vertical orientation. The contrast between the DC properties of the virus protein and the DNA stored within the nanogaps is clearly illustrated in Fig. 11, as demonstrated by ID-VGS [26]. Features such as ION, Vth, SS, and ION/IOFF are encompassed within this particular category. Fig. 11 depicts the changes that occur in SS and ION/IOFF based on the specific value of k under consideration. The variable marked by K replaces S-protein. As the value of k increases, there is an observed increase of around 20 % in the ratio of ION to IOFF, while the ratio of SS decreases by a factor of 2 % [26]. The occurrence of this phenomena does not exhibit any association with the quantity of k.

**Fig. 10:** VTFET-based biosensor's drain current sensitivity for unbiased charged biomolecules, b. Time-dependent response for k = 8.46 dielectric constant.

**Fig. 11:** Changes in the sub-threshold swing (SS) and the ION/IOFF at different levels of k for S-protein and C-DNA.

### 4.2 DNA charge density sensitivity analysis

The process of virus identification necessitates the conversion of viral RNA into DNA through the action of an enzyme called reverse transcriptase. The initial stage of the detecting process is being undertaken. Subsequently, the extracted DNA might be employed for investigating various viruses. The sensitivity of the sensor can be influenced by the density of charges present in DNA molecules. This phenomenon is feasible due to the potential for DNA molecules to encode information. The transportation of charges by DNA molecules renders this occurrence plausible. In this phase of the investigation, we assess the operational efficiency of the proposed sensor when exposed to DNA molecules with both positive and negative charges that have been immobilized within nanogaps. This evaluates the sensor's performance in this condition. Fig. 12a shows the drain current variance between DNA's greatest negative and positive charge densities during modelling. These two numbers will be compared. The transfer characteristics assume that DNA molecules occupy the nanogaps with k = 6.33. Fig. 12b shows transfer characteristics on a linear scale to explain current-charge density relationships. The linear scale has logarithmic characteristics.

**Fig. 12:** a Changes in transfer characteristics at different DNA charge densities when drain current is measured logarithmically, and b. Plot linearly.

The reverse transcriptase process facilitates the conversion of viral RNA into viral DNA, enabling its subsequent application in virus detection. The customization of sensor sensitivities can be achieved by modifying the charge density carried by DNA molecules. During this phase of the experiment, the proposed sensor undergoes rigorous testing by being subjected to immobilized nanogaps that contain DNA molecules with both positive and negative charges. Fig. 12a shows drain current modelling findings between DNA charge density extremes. The transfer properties are graphed assuming k = 6.33 DNA molecules occupy the nanogaps. Fig. 12b shows transfer characteristics on a linear scale, clarifying the current-charge density relationship.

(3) $$S\text{ensitivity}=Sensitivity\;\left(S_{N}\right)=V_{T,K-1}-\;V_{T,K}$$

Where $V_{T,K-1}$ and $V_{T,K}$ are the V_th_ of the ID–VGS characteristics for empty nanogaps and filled nanogaps, respectively. Fig. 13a displays a graphical representation of the ID-VGS properties of the sensor under investigation at k values of 1.2, 2.84, 6.33, and 8.46. The negative charge density, denoted as N bio, is held constant at N _bio_ = 1×108Ccm2. A rightward shift in the drain current is observed when the concentration of negatively charged DNA molecules exceeds the neutral value of −3 ×108Ccm2. The variance in Vth for the range of k examined in this investigation is depicted in Fig. 13b. Nevertheless, when the density of charged DNA remains constant, the value of Vth decreases as K grows. The determination of drain current sensitivity can be achieved by employing Equation (2). According to Fig. 13c, a rise in the concentrations of negative charge in DNA molecules is associated with a decrease in sensitivity.

**Fig. 13:** a. The transfer characteristics of a VTFET sensor for the detection of SARS-CoV-2 at a temperature of −1.9 × 10^12 C/cm2. B. The voltage at which DNA reaches its threshold (VT) in relation to concentrations of negative charge. C. The relationship between the negative charge density (Sn) of DNA and its sensitivity.

The decline in sensor sensitivity can be linked to the degradation of the drain current, which is caused by the drop in WS. Increasing the value of k leads to an increase in WS, hence causing a higher drain current and subsequently resulting in a greater level of sensitivity, assuming that VGS and –N remain constant. This clarifies the cause behind the correlation between a larger k number and an increased Sn. Consequently, the value of Vth will exhibit an increase when compared to that of biomolecules with neutral charges, as a higher gate voltage will be necessary to effectively clear the channel (see Fig. 13b). In a similar vein, Fig. 14 examines the influence of positively charged DNA on the sensor's output. Fig. 14a depicts the ID-VGS characteristics of the sensor under consideration, where N_bio_ is equal to N_bio_ = 1×108Ccm2, for various values of k, namely 1.2, 2.84, 6.33, and 8.46. According to Fig. 14b, an increase in positive charge density leads to a drop in Vth. The reason for this phenomenon is because an augmentation in the positive charge density, as represented by the equation q_N_/C_eff_ in Equation (4), leads to a corresponding elevation in the surface potential (WS). Consequently, this elevates the value of VGS. Consequently, the sensor will see a rise in channel conductance. Fig. 14c demonstrates that a higher concentration of positive charges in DNA leads to a device with greater sensitivity. The graph serves as evidence for this.

**Fig. 14:** a The transfer properties of a VTFET sensor at a DNA charge density of 1.9 × 10^12 C/cm2, the relationship between threshold voltage (VT) and various DNA charge densities, and the sensitivity (Sn) with respect to different DNA charge densities were investigated for the purpose of detecting SARS-CoV-2.

### 4.3 The impact of noise on the scalability of a TFET-based biosensor

Interface trap charges (ITCs) are a specific category of physical faults that have the potential to diminish the reliability of semiconductor devices. The model should incorporate models that account for the trap's capacity and the amount of charge it has stored. In this analysis, we delve deeper into the interface traps of the acceptor type. This particular type of trap has the capacity to retain a charge equivalent to that of a single electron, even though it lacks any charge when it is empty. Research is being conducted on uniform and Gaussian distributions.

Uniform: $N_{o};for\;E_{o}-0.5E_{s}<E<E_{o}+0.7E_{s}$.

(4) $$G_{s}=No\;\mathrm{Exp}\left(\;-\;\frac{E-E_{o}^{2}}{2E_{3}^{2}}\right)$$

In this particular scenario, the variables Energy Mid and Energy Sig are utilized to express values in electron volts (eV) for E0 (zero eV) and ES (tenths of a volt), respectively. Meanwhile, N0 remains constant at a trap concentration of 1×108Ccm2. Fig. 15a displays the charge density distributions in the traps as a function of energy, providing a visual representation of the data. Fig. 15b depicts the impact of ITCs on the transfer characteristics of the VTFET biosensor, as seen in the curves. The diminished drain current can be mostly attributed to the presence of traps in close proximity at the junction of tunnelling. The findings are depicted in Fig. 15a presented below. Fig. 15b illustrates the alteration of transfer attribute curves in VTFET biosensors upon the addition of ITCs. The curves are well exhibited by biosensors. The primary factor contributing to the reduction in drain current is the presence of adjacent traps at the tunnelling joint. The stochastic capture and subsequent release of carriers constitutes a fundamental factor influencing the overall quantity of carriers available for contemporary transportation.

**Fig. 15:** a The relationship between trap charge density and energy, as well as the impact of trap distributions of uniform and Gaussian types on drain current characteristics.

The confined charges possess the capacity to disrupt both the spatial arrangement of the carriers and the electric field. The researchers exhibit a specific interest in the auditory emissions generated by these traps. The presence of this specific form of noise is inherently interconnected with the operational principles of the device and cannot be entirely eradicated. Therefore, it is imperative to minimize it by meticulously choosing the material and shape of the gadget. The link between frequency and noise at 1 MHz and 10 GHz may be shown in Fig. 16a and b, illustrating the impact of increasing the pocket length on the noise spectral density (Sid) of the drain current. Furthermore, Fig. 16c illustrates the distribution of net Sid as a function of frequency. The value of Sid reaches its maximum at lower frequencies and decreases to its minimum at higher frequencies. The noise in question is commonly known as low-frequency noise due to its relatively low frequency. The Net Sid value is greater when L _Pocket_ is 10 nm compared to L Pocket values of 15 nm or 20 nm. Considering this, a value of L _Pocket_ = 20 nm is incorporated into any analysis to account for both noise and drain current.

**Fig. 16:** a. The spectrum density of the noise in the drain current of a TFET-based biosensor at a. f = 1 MHz b. f = 10 GHz, c. Net Sid w.r.t. frequency.

Fig. 17a illustrates the differences in sensitivity that occur when traps are used compared to when they are not employed. Although the inclusion of traps leads to a notable reduction in sensitivity, it remains sufficiently high to surpass the performance of the most sensitive biosensors presently available in the market. The lower limit of detection (LOD), often referred to as the detection threshold, is determined by the signal-to-noise ratio (SNR), which is obtained by the I–V characterization of the noise. The expression of the signal-to-noise ratio (SNR) for bio-FET devices can be represented using the number fluctuation model.

(5) $$SNR=\frac{G_{m}}{\sqrt{S_{ID}}}=\frac{G_{m}}{\sqrt{S_{VFB}}}$$

**Fig. 17:** a. The sensitivity of a VTFET-based biosensor is measured at k = 12. B, both with and without traps. SNR plotted against solution gate voltage, c Comparing the simulation and experimental results of the biosensor.

The lower limit of the Line-of-Sight (LOD) is established by the ratio of the flat-band voltage variations generated by traps and interface states to the signal-to-noise ratio (1/SNR). This lower limitation might be regarded as the upper limit. Fig. 17b illustrates the correlation between the signal-to-noise ratio and the voltage applied to the solution gate. A maximum signal-to-noise ratio of 10,050 was attained, indicating a minimum detectable voltage of *90. The point at which the highest transconductance is seen is gm, which represents the best signal-to-noise ratio. The limit of detection (LOD) is significantly reduced due to the exceptionally low minimum detectable voltage. The sensitivity of the created biosensor is compared between the simulated and experimental data, revealing significant findings. These results are illustrated in Fig. 17c.

## 5 Next‐generation sequencing

An analysis is conducted on the full genome sequencing data obtained from samples that exhibited positive results for SARS-CoV-2. Upon completion of the analysis, the mutation profile of these samples is shown. Based on the data we obtained [[25], [26], [27]], we present a summary of the mutation pattern of the genomes and the distribution of clades among the isolates, considering their genomic diversity. The present analysis is predicated by the genetic diversity exhibited by the isolates.

### 5.1 Data analysis

A total of fifty samples were supplied by patients to the medical facility, consisting of thirty male samples and twenty female samples. The age range of the patients in the study spanned from one to seventy, with a mean age of thirty-five for the entire group. All patients exhibited positive results for SARSCoV2 in their respective tests, as indicated by Ct values below twenty. The study's samples were initially obtained from individuals who were suspected to be currently infected with SARS-CoV2 at the time of sample collection. This decision was made as part of the regular diagnostic procedures that are implemented. After the samples were collected, they were transported to the laboratory and stored at a temperature of 4 °C until the analytical results were obtained. The samples were subjected to examination using the Bio Speedy SARSCoV2 (2019nCoV) qPCR Detection Kit v5.3, which was produced by Bioeksen, prior to the sequencing procedure. Prior to the sequencing of the samples, this procedure was conducted. The technique was completed prior to cooling the samples at a temperature of 80 °C. Samples with high viral loads and Ct values below 20 were selected in order to mitigate the adverse impacts of the buffer used for extracting viral nucleic acid in transfer tubes. This buffer is known to cause RNA degradation and subsequent loss of nucleic acid. The matter at hand has great importance due to the requirement of a considerable viral load in order to achieve optimal performance in next-generation sequencing (NGS). The purpose of this study was to employ Next-Generation Sequencing (NGS) technology for the analysis of the samples. The samples could only be kept for a prolonged period of time in transfer tubes that contained a buffer for the extraction of viral nucleic acid.

Consequently, the nucleic acid composition of the samples exhibited a progressive decline during the duration of our investigation. Consequently, we opted to exclusively employ fresh samples that had undergone recent processing in our laboratory, as we anticipated a higher likelihood of these samples containing significant amounts of virus. To obtain pertinent outcomes using Next-Generation Sequencing (NGS), a substantial quantity of viral material with high-quality nucleic acid is required. It was hypothesized that using samples with a high viral load will facilitate the production of high-quality PCR products and enhance the quality of data generated by NGS. There exists empirical data indicating a positive correlation between elevated viral loads and heightened levels of infectivity and severity of sickness [27]. This finding provides an additional rationale for selecting samples characterized by high viral loads. Based on the results, samples with elevated amounts of the virus were chosen.

Initially, our inquiry did not include a comprehensive analysis and comparison of mutations observed in patients with diverse age groups, genders, or levels of disease manifestation. The objective of this investigation was to determine the presence or absence of a mutation in the samples collected from our prospective patients. Given these concerns, we have developed a working hypothesis that posits the ability to differentiate mutations in samples derived from individuals exhibiting very elevated viral loads. Our hypothesis posited that we would possess the capability to identify mutations in samples derived from individuals diagnosed with HIV.

The procedure of constructing an NGS library consisted of four distinct stages, wherein the SARS-CoV-2 Panel and Dual-Indexed PCR Primers were employed as the primary components. As part of the Global Initiative on Sharing All Influenza Data (GISAID), the classification of the clade responsible for severe acute respiratory syndrome–coronavirus 2 (SARS–CoV2) was supplied by the national agency in India. The technique developed by GISAID involves the identification of significant clades through the analysis of alterations in specific markers within eight primary phylogenetic groups. As a consequence, the system was ultimately developed. The SARS-CoV-2 sequences presented in GISAID from India derive from a wide range of clades. The demultiplexed FASTQ files were cleaned and the adapter sequences were eliminated using version 3.0 of Cutadapt. Subsequently, the Genome Detective Virus Tool was employed to do 15 further data analysis on the pre-sequencing cleaned and trimmed data. The Genomics Analyzer Virus Tool is an online software that carries out several activities on Next-Generation Sequencing (NGS) data, including analyzing the quality of reads, eliminating reads, mapping reads, assembling reads, and generating consensus sequences. These routines are executed on the Next-Generation Sequencing (NGS) data [27,28]. Assembly sequences exhibiting a significant amount of missing data, divergence, or ambiguous nucleotides were excluded from further analysis. An assessment of the consensus sequence's quality was conducted using a diverse range of metrics. The Nextclade tool was utilized to evaluate both sequencing mistakes and assembly quality.

### 5.2 Mutational dimension

A grand total of 600 unique modifications were detected, with only 250 of those being completely original. Out of the total 250 possible mutations (245 substitutions and 5 deletions), just one instance of each of the remaining 200 mutations was seen in any of the sequences. A cumulative count of 250 distinct mutations has been ascertained, comprising 15 instances observed in noncoding regions, 5 instances involving deletions, and the remaining 150 instances categorized as missense mutations. It is crucial to emphasize the potentially substantial functional implications that mutations in these particular gene regions may have within the domain of vaccine development and other therapeutic approaches [29].

### 5.3 GISAID and next strain clade distribution

Three separate GISAID clades emerge when the sequences are clustered using the GISAID approach. Among the 35 sequences examined, 10 were classified within the G clade, 20 within the GR clade, and 5 within the GH clade. The Next strain sequences were found to consist of two primary clades.

### 5.4 Discussion on mutational dimension

There exists empirical data indicating that the mutations resulting from this evolutionary process have exerted an influence on the virulence of the virus. From the onset of the SARS pandemic, the genome of SARS-CoV-2 has undergone rapid evolutionary changes. Due to the widespread accessibility of NGS technologies, mutations and variants are regularly monitored, and a vast number of complete genomes can be freely downloaded from the internet.

The observation of approximately 3000 distinct point mutations in virus isolates obtained globally provides evidence supporting the notion that the occurrence of genetic alterations has escalated during the pandemic. The aforementioned finding was a direct result of the identification of over three thousand distinct virus isolates. A study of 160 genomes reveals that Indian SARS-CoV-2 isolates exhibit a greater mutation rate, aligning with findings reported globally. This information aligns with the findings reported on an international scale. Research conducted in the past has indicated that the regions of the genome harbouring the genes S and RdRp exhibit the most pronounced mutation rates. The sequences we have obtained exhibit a significant frequency of missense mutations, which align with the findings of earlier studies conducted in several regions, including Asia. Many of these modifications commonly take place in gene areas that are linked to the production of enzymes and cofactors, both of which play a crucial role in the replication of the SARS-CoV2 genome. The present study aimed to examine the potential consequences of commonly occurring mutations in the sequences, considering their genomic placements. However, an analysis of the changes in protein structure and functional assessments of these mutations was not conducted. We focused mostly on the sequences alone and the possible alterations that could occur within them. According to the results of the mutation study [28,29], it was observed that all of the sequences under investigation revealed the D614G mutation in the spike glycoprotein (23403 A > G), as well as the P323L mutation in the nsp12/RdRp (14408C > T).

Previous studies have provided evidence indicating a greater probability of individuals of Asian descent possessing both of these mutations simultaneously within their genomes. Throughout the course of the pandemic, the D614G mutation gradually emerged as the dominant variant across all geographical regions worldwide. People with the D614G mutation have increased levels of viruses in their bodies. The virus is capable of adhering to the host cell and subsequently infiltrating the cell via a protein known as the spike. Similarly, a study done in India yielded same results. The aforementioned research was conducted at that location. Recent research has established a correlation between the D614G and P323L mutations observed in SARS-CoV-2 with the occurrence of more severe cases of COVID-19. The 241C > T mutation, which is highly widespread in the 5′UTR of SARSCoV2, was present in all of our sequences [29,30]. Sample 10 had a distinct mutation (24545 A > G; R995G) in its spike protein sequence, while Sample 15 displayed a novel mutation (24763G > C; V1068L) in its spike protein sequence. The S2 domain of the protein has undergone two changes. Modifying the S2 domain, a viral fusion peptide, can increase infectivity by improving fusion activity and enhancing the stability of membrane fusion. The rationale behind this phenomenon is that the S2 domain functions as a peptide for the purpose of viral fusion. The diagram [30] provides a visual depiction of the categorization of the garment and its prevalence throughout the Covid-19 era.

## 6 Conclusion

The analysis of the spike, envelope, and DNA proteins of the SARS-CoV-2 virus will be conducted using a biosensor that incorporates a vertical tunnel field-effect transistor (VTFET). The primary objective in the creation of the biosensor was to assess its ability to accurately detect the specific medication present in clinical samples. The sensitivity of the proposed sensor was assessed by quantifying the alteration in the drain current, enabling an examination of the sensor's dynamic range. The depiction of the hybridized biomolecules located within the nanogaps is provided by the dielectric constant equivalent of the viral proteins. The sensitivity of the proposed sensor has been determined to be roughly 115, suggesting its potential as a sensing tool of excellent quality. This observation demonstrates the sensor's ability to operate as a high-quality sensing tool. To detect changes that modify the ability of SARS-CoV-2 to spread and cause disease, we do sensitivity analysis on the density of electrically charged DNA and analyze the entire genomes of the virus. Our objective is to ascertain these modifications. This study primarily aimed to investigate the monitoring of mutations and their impact on virulence variables, including resistance to host cell receptors, viral load, and mortality. The field of genomic epidemiology, comprised of the sequencing of the viral genome, exhibits promise in enhancing comprehension of transmission mechanisms and evaluating novel preventive strategies.

## Ethical approval (human ethics and consent to participate required for this manuscript)

Not Applicable.

## Availability of data and materials

The data can be available based on the request from the authors.

## CRediT authorship contribution statement

**M. Venkatesh:** Visualization, Validation, Software, Resources, Methodology, Data curation. **P. Parthasarathy:** Writing – review & editing, Writing – original draft, Validation, Supervision, Project administration, Formal analysis, Data curation, Conceptualization.

## Declaration of competing interest

The authors declare that they have no known competing financial interests or personal relationships that could have appeared to influence the work reported in this paper.
